The article "Texture Features of Computed Tomography Image under the Artificial Intelligence Algorithm and Its Predictive Value for Colorectal Liver Metastasis" was published in 2022. Journal: Contrast Media Mol Imaging.

# Texture Features of Computed Tomography Image under the Artificial Intelligence Algorithm and Its Predictive Value for Colorectal Liver Metastasis

**DOI:** 10.1155/2022/2279018

**Published:** 2022-07-19

**Authors:** Derong Sun, Jianjiang Dong, Yindong Mu, Fangwei Li

**Affiliations:** ^1^Department of Gastroenterology, The Fourth Hospital of Harbin Medical University, Harbin 150001, China; ^2^Department of Histology and Embryology, Mudanjiang Medical University, Mudanjiang 157011, China; ^3^Department of Nuclear Medicine, Affiliated Hongqi Hospital of Mudanjiang Medical University, Mudanjiang 157011, China

## Abstract

The aim of this research was to investigate the predictive role of texture features in computed tomography (CT) images based on artificial intelligence (AI) algorithms for colorectal liver metastases (CRLM). A total of 150 patients with colorectal cancer who were admitted to the hospital were selected as the research objects and randomly divided into three groups with 50 cases in each group. The patients who were found to suffer from the CRLM in the initial examination were included in group A. Patients who were found with CRLM in the follow-up were assigned to group B (B1: metastasis within 0.5 years, 16 cases; B2: metastasis within 0.5–1.0 years, 17 cases; and B3: metastasis within 1.0–2.0 years, 17 cases). Patients without liver metastases during the initial examination and subsequent follow-up were designated as group C. Image textures were analyzed for patients in each group. The prediction accuracy, sensitivity, and specificity of CRLM in patients with six classifiers were calculated, based on which the receiver operator characteristic (ROC) curves were drawn. The results showed that the logistic regression (LR) classifier had the highest prediction accuracy, sensitivity, and specificity, showing the best prediction effect, followed by the linear discriminant (LD) classifier. The prediction accuracy, sensitivity, and specificity of the LR classifier were higher in group B1 and group B3, and the prediction effect was better than that in group B2. The texture features of CT images based on the AI algorithms showed a good prediction effect on CRLM and had a guiding significance for the early diagnosis and treatment of CRLM. In addition, the LR classifier showed the best prediction effect and high clinical value and can be popularized and applied.

## 1. Introduction

Colorectal cancer is a common cancer and ranks third among common malignant tumors with a high mortality rate [1]. Most colorectal cancer patients experience constipation, and some suffer from diarrhea, often alternating between the two. Intestinal obstruction may occur in the late stage of the patient, which affects the patient's digestion, causes anemia and weight loss, and sharply deteriorates physical fitness, which increases the difficulty of treatment [2–4]. The early detection of the colorectal cancer is difficult, and the early symptoms are not obvious so that the patient's attention is not attracted. After the symptoms are obvious, the disease has developed to a deeper degree, and the prognosis is poor [5, 6]. Colorectal cancer patients often develop liver metastasis, which will aggravate the patient's condition and threaten the patient's life safety [7]. The liver is most prone to metastases in colorectal cancer patients, and the treatment of colorectal liver metastasis (CRLM) is difficult, the disease risk of patients is high, and the mortality rate is greatly increased. Generally, patients with CRLM require surgical treatment, but patients generally cannot meet the standard of surgical resection when the disease is discovered. Therefore, the prediction and early treatment of colorectal cancer patients are extremely important for the prognosis of patients [8–10].

The gold standard for the diagnosis of colorectal cancer is pathology, and imaging methods play an important role in disease diagnosis, pretreatment assessment of lesion extent, and prognosis monitoring [11]. Imaging examination has a certain predictive effect on tumor location, size, shape, extent of invasion, and the presence of distant metastasis and has a high clinical value [12, 13]. Image texture analysis is a new type of image processing technology in recent years. It obtains relevant parameters by analyzing images and has positive significance in the judgment and analysis of computed tomography (CT) images [14, 15]. Texture analysis quantifies tissue heterogeneity by evaluating the texture roughness and distribution within the lesion, and it can evaluate the characteristics of the lesion in more detail, which is helpful for judging the characteristics of the tumor and evaluating the prognosis and metastasis [16, 17]. Analyzing whether texture parameters correlate with disease metastases requires modeling. The commonly used modeling methods are logistic regression (LR), linear discriminant (LD), k-nearest-neighbor (KNN), naive Bayesian (NB), decision tree (DT), support vector machine (SVM), etc. [18–20]. In this work, all these six classifiers were used to explore the prediction effect of CRLM and analyze the predictive value of CT image texture features analysis for CRLM.

This work explored the predictive effect of CT image texture features based on artificial intelligence (AI) algorithms on CRLM. The research objects were examined by CT, the CT images were processed and analyzed, and image texture analysis was performed. The prediction accuracy, sensitivity, and specificity of CRLM under the conditions of six classifiers for different groups of patients were calculated, and the prediction effects of the six classifiers for image texture analysis were analyzed. It was expected to provide a clinical guidance for CT image processing and analysis of colorectal cancer patients and offers a reference for liver metastasis prediction and early treatment of colorectal cancer patients.

## 2. Materials and Methods

### 2.1. Research Objects

In this research, 150 patients with colorectal cancer admitted to the hospital from January 2020 to December 2021 were selected as the research objects and divided into three groups. Among them, 50 patients in group A were found to have CRLM during the initial examination; 50 patients in group B were found to have CRLM in subsequent follow-up imaging; and 50 patients in group C were found to have no CRLM in the initial examination and follow-up. Among them, the patients in group B were further rolled into group B1, group B2, and group B3. The patients in group B1 were found to have CRLM within six months, with a total of 16 cases. The 17 patients in group B2 were found with CRLM within six months to one year, and there were 17 patients in group B3, who were found with CRLM within one to two years. The objects included were subjected to CT examination, and the prediction effect of the CT image texture feature analysis of the AI algorithm on CRLM was analyzed. This research had been approved by the ethics committee of the hospital.

Inclusion criteria were patients with complete medical records and imaging data; patients with no other vital organ diseases; patients with no central nervous system diseases, endocrine system diseases, and other serious physical diseases; patients with no communication barriers; and patients who signed informed consents.

Exclusion criteria were patients who underwent radiotherapy, chemotherapy or radiotherapy, and chemotherapy before CT examination; patients had intestinal inflammation, infection, and other diseases; patients who were pregnant or lactating women; and patients unwilling to participate in this experiment.

### 2.2. CT

All patients were examined with a 64-slice spiral CT system. The tube voltage was 120 kV, the tube current was 260 mA, the substrate was 512 × 512, the scanning slice thickness was 5 mm, and the slice interval was 5 mm. The contrast agent iohexol was injected into the cubital vein with a high pressure syringe at a flow rate of 3.0 mL/s for a total dose of less than or equal to 90 mL. The scanning time of the arterial phase was 20 s, and the portal venous phase was collected 30–33 s after the arterial phase. Delayed scans were performed three minutes after administration of the contrast agent. The reconstructed slices were 3 mm thick and 3 mm apart. The scanning range was from the top of the skull to the proximal femur.

### 2.3. Image Processing and Analysis

#### 2.3.1. Lesion Segmentation

The region of interest (ROI) was delineated manually on CT images of colorectal cancer primary lesions, and lesions were segmented. It should keep a distance of 2–3 mm from the tumor edge to delineate the ROI, avoid the calcified, necrotic cystic part of the lesion, and include the solid part of the lesion in the ROI.

#### 2.3.2. Texture Analysis

After lesion segmentation, texture features were calculated and extracted. The texture parameters can be obtained by using a grayscale histogram, a grayscale cooccurrence matrix, or the like. The data are dimensionally reduced by methods such as the rank sum test (ANOWA + MW), correlation analysis, and Lasso, using LR, LD, KNN, NB, DT, and SVM classifiers classify the extracted texture features. In addition, it should calculate the accuracy, sensitivity, and specificity of each classifier's predictions to arrive at the optimal classification model.

### 2.4. Observation Indicators

The general data of the two groups of patients were compared, including gender, age, years of education, medical history, T stage, N stage, M stage, and carcinoembryonic antigen (CEA). T (for tumor): the size of the primary tumor. N (for regional lymph nodes): the number of cancers that have spread to nearby regional lymph nodes. M (for distant metastasis): the cancer has spread to distant parts of the body. TNM staging had been confirmed by pathological examination.

The accuracy, sensitivity, and specificity of predicting CRLM under six classifiers for patients in different groups were calculated. Equations (1)–(3) showed the calculation methods of sensitivity, specificity, and accuracy, respectively. Among them, PB referred to the number of patients predicted to be CRLM, PM was the number of patients with CRLM in the examination result, DB represented the number of patients predicted to be without CRLM, and DM was the number of patients with no CRLM in the examination result.

(1) $$\begin{array}{c} \mathrm{Sensitivity=}\frac{\mathrm{DM}}{\mathrm{PM}}, \end{array}$$

(2) $$\begin{array}{c} \mathrm{Specificity=}\frac{\mathrm{DB}}{\mathrm{PB}}, \end{array}$$

(3) $$\begin{array}{c} \mathrm{Accuracy=}\frac{\mathrm{DM+DB}}{\mathrm{PB+PM}}. \end{array}$$

In addition, it should draw the ROC curves of predicted CRLM under the six classifiers of patients in group A, B, and C and the ROC curves of predicted CRLM under the LR classifier of patients in groups B1, B2, and B3.

### 2.5. Statistical Analysis

Excel 2016 was used to record and summarize data. SPSS 20.0 was used for data statistics and analysis. The mean ± standard deviation (*X* ± *S*) represented the measurement data, and the *t* test was used. Percentage (%) was the representation of count data, using the *X*^2^ test. *P* < 0.05 was considered statistically significant.

## 3. Results

### 3.1. Comparison of General Data

The general data of the three groups of patients were shown in Table 1. There were no statistical differences in gender, age, years of education, and medical history among the three groups of patients, so they were comparable.

Figure 1 showed the comparison of the general data of the three groups of patients, where Figure 1(a) compared T stage, Figure 1(b) compared N stage, Figure 1(c) compared M stage, and Figure 1(d) compared CEA. In group A, there were 0 TI patients, 0 T2 patients, 20 T3 patients, 30 T4 patients, 18 N0 patients, 32 N1-2 patients, 0 M0 patients, 50 M1 patients, 9 patients with CEA < 5 mcg/L, and 41 patients with CEA ≥ 5 mcg/L. In group B, there were 0 patients with TI, 2 patients with T2, 19 patients with T3, 29 patients with T4, 13 patients with N0, 37 patients with N1-2, 50 patients with M0, 0 patients with M1, 15 patients with CEA < 5 mcg/L, and 35 patients with CEA ≥ 5 mcg/L. In group C, there were 0 patients with TI, 4 patients with T2, 9 patients with T3, 37 patients with T4, 36 patients with N0, 14 patients with N1-2, 50 patients with M0, 0 patients with M1, 23 patients with CEA < 5 mcg/L, and 27 patients with CEA ≥5 mcg/L.

### 3.2. CT Image Analysis and ROI Delineation of Primary Tumor

Figure 2 showed CT image analysis and ROI delineation of the primary tumor in a colorectal cancer patient. Among them, Figure 2(a) was the CT image of a patient with colorectal cancer, Figure 2(b) was the patient's manual delineation of the lesion site, the patient's lesion area was a red dashed circle, and Figure 2(c) was the drawn lesion ROI. It showed that after a CT scan of the patient, a large tumor, about 8 cm by 5 cm in size, was found in the colon.

### 3.3. Prediction Accuracy of Six Classifiers

Figure 3 showed the prediction accuracy performance of the six classifiers for the three groups of patients, where Figures 3(a)–3(c) showed the accuracy, sensitivity, and specificity, respectively. The prediction accuracy of the LR classifier for patients in group A was 0.78, the sensitivity was 0.74, and the specificity was 0.77. The prediction accuracy of the LR classifier for patients in group B was 0.77, the sensitivity was 0.81, and the specificity was 0.76. The prediction accuracy of the LR classifier for group C patients was 0.76, the sensitivity was 0.78, and the specificity was 0.78. The prediction accuracy results of the six classifiers for the three groups of patients showed that the LR classifier had the best prediction effect, which was significantly better than other classifiers, followed by the LD classifier.

### 3.4. The ROC Curves of Six Classifiers Predicting CRLM in Three Groups of Patients

Figures 4–6 were the ROC curves of the six classifiers predicting the CRLM of the three groups of patients. The prediction effect of the patients in group A was better than that in groups B and C. Among the six classifiers, the LR classifier and LD classifier had the best prediction effect, the KNN classifier and DT classifier had the worst prediction effect, and the LR classifier had a great advantage in predicting CRLM of patients.

### 3.5. The Effect of the LR Classifier in Predicting CRLM in Group B Patients

Figure 7 showed the effect of the LR classifier on predicting CRLM in patients in group B, where Figures 7(a)–7(c) showed accuracy, sensitivity, and specificity, respectively. The prediction accuracy of the LR classifier for patients in group B1 was 0.78, the sensitivity was 0.72, and the specificity was 0.77. The prediction accuracy of the LR classifier for patients in group B2 was 0.75, the sensitivity was 0.70, and the specificity was 0.73. The prediction accuracy of the LR classification for patients in group B3 was 0.77, the sensitivity was 0.73, and the specificity was 0.76. The effect of the LR classifier in predicting CRLM of patients in B1 and B3 groups was significantly better than that of patients in B2 group (*P* < 0.05).

### 3.6. ROC Curve of LR Classifier Predicting CRLM of Patients in Group B

Figure 8 showed the ROC curve of the LR classifier predicting the CRLM of patients in group B. It revealed that the effect of the LR classifier in predicting CRLM of patients in groups B1 and B3 was significantly better than that of patients in group B2 and had a better prediction effect.

## 4. Discussion

Colorectal cancer is very common in malignant tumors, with a high metastasis rate and high fatality rate, which seriously threatens the life safety of patients [21]. Patients usually have a series of digestive tract symptoms, which make the patient's constitution worse, and the prognosis is poor. Many systemic symptoms will appear in the later stage, which will bring pain to the patient and increase the difficulty in the treatment of the disease [22]. Colorectal cancer patients have a high probability of liver metastases, and liver metastases will aggravate the disease and increase the mortality of patients [23]. Early prediction and diagnosis of CRLM in patients is extremely important for the patient's prognosis. Early detection and treatment are an important way to control and treat the disease. Early prediction of the disease can give colorectal cancer patients intervention before the disease aggravates and spreads, improving the prognosis and increasing the patient's life span [24]. Accurate prediction of liver metastasis in colorectal cancer patients is an important measure to promote patients to receive treatment as soon as possible. Therefore, it is extremely important to explore the prediction method of liver metastasis in colorectal cancer patients, which has become a research hotspot in clinical practice [25].

Imaging examination has become the routine examination of colorectal cancer patients at present, which is superior to other examination methods and is the preferred diagnostic technology for colorectal cancer patients. It is a noninvasive examination method, which can significantly reduce the discomfort of patients and has high safety [26]. Texture analysis can quantify the intuitive quality described by terms such as roughness, smoothness, or bump as a function of spatial variation in pixel intensity. The heterogeneity of different results can be explored through texture analysis to identify texture features that can be used for diagnosis and prediction [27]. At present, texture analysis has been widely used in tumor imaging, has important value in the judgment of benign and malignant tumors, metastasis, and prognosis, and can guide clinical treatment. Zheng et al. [28] explored the application of a combined model based on clinical and enhanced CT texture features in predicting liver metastases from high-risk gastrointestinal stromal tumors (GISTs) and found that texture-based radiomic features of portal venous phase CT images could noninvasively predict liver metastases in high-risk gastrointestinal stromal tumors, and integrating other clinical variables into the model could further improve liver metastasis risk prediction. Granata et al. [29] analyzed the efficacy of radiomics signatures obtained from arterial and portal vein MRI in predicting the clinical outcome in patients with colorectal liver metastases, assessing recurrence, mutational status, pathological features (mucinous and tumor budding), and surgical resection margins; it was found that identifying tumor budding using the 11 texture features extracted by the KNN classifier yielded the best results with 95% accuracy, 84% sensitivity, and 99% specificity.

In this work, the prediction effect of CT image texture features based on AI algorithms on CRLM was analyzed. Image texture analysis was performed on three groups of patients, the prediction accuracy, sensitivity, and specificity of CRLM in three groups of patients under six classifier conditions were calculated, and the ROC curves of CRLM prediction were plotted. The results of the work showed that the prediction accuracy of the LR classifier was 0.78 in group A, 0.77 in group B, and 0.76 in group C, and the sensitivity of LR classifier prediction in group A was 0.74, 0.81 in group B, and 0.78 in group C, and the specificity predicted by the LR classifier was 0.77 in group A, 0.76 in group B, and 0.78 in group C. The prediction accuracy, sensitivity, and specificity of LR classifier were the highest, and the prediction effect was the best, followed by the LD classifier. The accuracy of LR classifier prediction was 0.78 for patients in group B1, 0.75 for group B2, and 0.77 for group B3; the sensitivity of LR classifier prediction for patients was 0.72 in group B1, 0.70 in group B2, and 0.73 in group B3. The specificity predicted by the LR classifier was 0.77 in group B1, 0.73 in B2 group, and 0.76 in group B3. The accuracy, sensitivity, and specificity of LR classifier prediction were higher in group B1 and group B3, and the prediction effect was better than that in group B2. The analysis of CT imaging texture features can be applied to the prediction of CRLM patients, which has guiding significance for the early diagnosis and treatment of CRLM of patients. The LR classifier has a good prediction effect and can be popularized and applied in clinical practice.

## 5. Conclusion

CT image texture features had important guiding significance for predicting liver metastases in colorectal cancer patients. The LR classifier had the best prediction effect and can provide a reference for the diagnosis and prediction of colorectal cancer patients, which had positive significance and can be popularized and applied in clinical practice. The disadvantage of this work was that the sample size was small, and further research and validation were needed.

## Figures and Tables

**Figure 1:** Comparison of general data of three groups of patients. (a) T stage, (b) N stage, (c) M stage, and (d) CEA.

**Figure 2:** CT image analysis and ROI delineation of primary lesions in patients with colorectal cancer. Case 1, male, 56 years old, CRLM. (a) CT image of a patient with colorectal cancer; (b) lesion manually drawn by the patient; (c) ROI of the drawn lesion.

**Figure 3:** Prediction accuracy performance of 6 classifiers for three groups of patients (a) accuracy, (b) sensitivity, and (c) specificity.

**Figure 4:** ROC curves of six classifiers predicting CRLM of patients in group A.

**Figure 5:** ROC curves of six classifiers predicting CRLM of patients in group B.

**Figure 6:** ROC curves of six classifiers predicting CRLM of patients in group C.

**Figure 7:** Prediction effect of the LR classifier on CRLM of patients in group B. (a): accuracy, (b): sensitivity, (c): specificity. ^*∗*^ compared with other groups, *P* < 0.05.

**Figure 8:** ROC curve of the LR classifier predicting CRLM of patients in group B.

**Table 1:** Comparison of general data of three groups of patients.

Group	Males/females	Age (years old)	Years of education (years)	Medical history (years)
Group A	31/19	51.37 ± 8.92	12.77 ± 2.35	6.17 ± 3.38
Group B	32/18	52.42 ± 8.77	12.65 ± 2.56	6.27 ± 3.24
Group C	30/20	51.79 ± 8.53	12.82 ± 2.39	6.97 ± 3.19

## Data Availability

The data used to support the findings of this study are available from the corresponding author upon request.
